The article "Combining autologous bone marrow buffy coat and angioconductive bioceramic rod grafting with advanced core decompression improves short-term outcomes in early avascular necrosis of the femoral head: a prospective, randomized, comparative study" was published in 2021. Journal: Stem Cell Res Ther.

# Combining autologous bone marrow buffy coat and angioconductive bioceramic rod grafting with advanced core decompression improves short-term outcomes in early avascular necrosis of the femoral head: a prospective, randomized, comparative study

**DOI:** 10.1186/s13287-021-02436-0

**Published:** 2021-06-19

**Authors:** Qingtian Li, Weihong Liao, Guangtao Fu, Junxing Liao, Ruiying Zhang, Mengyuan Li, Yuhui Yang, Yuanchen Ma, Minghao Zheng, Qiujian Zheng

**Affiliations:** 1 Department of Orthopedics, Guangdong Provincial People’s Hospital,Guangdong Academy of Medical Sciences, Guangzhou, Guangdong Province People’s Republic of China; 2 The Second School of Clinical Medicine, Southern Medical University, Guangzhou, People’s Republic of China; 3 Centre for Orthopaedic Translational Research, School of Surgery, The University of Western Australia, M Block, QE2 Medical Centre, Monash Ave, Nedlands, WA 6009 Australia

**Keywords:** Autologous bone marrow buffy coat, Angioconductive bioceramic rod, Advanced core decompression, Avascular necrosis of the femoral head

## Abstract

**Background:**

Treatment of avascular necrosis of the femoral head (ANFH) in young patients remains a clinical challenge. A current controversy is whether hip-preserving surgery results in better outcomes. The adverse effects of hip-preserving surgery are associated with the fill material for the necrotic areas. This study aims to evaluate the early effects of autologous bone marrow buffy coat (BBC) and angioconductive bioceramic rod (ABR) grafting with advanced core decompression (ACD) on early ANFH.

**Methods:**

Forty-four (57 hips) patients with early ANFH from 2015 to 2020 were recruited for this study. They were randomized into two groups: group A received ACD, BBC, and ABR grafting; group B received treatment of ACD with β-tricalcium phosphate (β-TCP) granules and ABR grafting. The outcomes were assessed using the Harris Hip Scores (HHS) and survival rate analysis. The follow-up endpoint was defined as conversion to total hip arthroplasty (THA).

**Results:**

Forty patients (51 hips) were ultimately included in this study for analysis. Compared with group B, patients in group A had higher postoperative function score (*P* = 0.032) and postoperative Harris Hip Scores (HHS) (*P* = 0.041). Kaplan-Meier analysis showed a trend that the survivorship of the femoral head was higher in group A than in group B.

**Conclusion:**

The short-term follow-up results showed that the autologous bone marrow buffy coat and angioconductive bioceramic rod grafting with advanced core decompression is effective in the treatment of early ANFH.

**Trial registration:**

Chictr.org.cn, ChiCTR2000039595. Retrospectively registered on 11 February 2015.

## Background

Avascular necrosis of the femoral head (ANFH) is a common, refractory disease with multiple etiologies including long-term use of glucocorticoids, alcohol abuse, and hip trauma [1, 2]. The disease often progresses and results in femoral head collapse and hip osteoarthritis over time [3]. Despite the excellent survivorship of total hip arthroplasty (THA), the majority of patients who receive THA surgery are young. Therefore, THA is not an optimal therapy for young patients with ANFH [4, 5]. Hip-preserving surgery for early ANFH can relieve joint pain, reconstruct joint function, and delay or avoid THA. Presently, hip-preserving surgery includes different methods such as core decompression (CD), femoral osteotomy, bone grafting (vascularized or non-vascularized), porous tantalum rod grafts, and cell-based therapy.

Accumulating evidence indicates that cell therapy, including bone mesenchymal stem cell (BMSC) and bone marrow concentrates containing bone marrow-derived cells, is beneficial in relieving pain, reducing time to collapse, and delaying or avoiding THA for end-stage ANFH [6–8]. We have reported the use of the autologous bone marrow aspirated buffy coat (BBC) combined with core decompression (CD) for the treatment of osteonecrosis of femoral head [9]. Our randomized control study showed consistent improvement in pain relief delays the progression of pathological stage. The 10-year follow-up showed that the use of autologous BBC in combination with core decompression is more effective than the use of core decompression alone. Based on our previous studies showing that combining cell therapy with other treatment modalities can achieve better clinical outcome, we asked the question if combining BBC with bioceramic material can also achieve a similar outcome. The bioceramic materials used in this study include dense β-TCP granules (diameter 1.0–3.0 mm, no microporosity), porous β-TCP granules (diameter 1.0–3.5 mm, macropore 500–600 μm, interconnection 120 μm), and porous bioceramic rods (diameter 10 mm, length 80 mm, macropore 500–600 μm, interconnection 120 μm) (Bio-Lu, 201114, Shanghai, China).

The angioconductive bioceramic rod (ABR) has recently gained popularity for the treatment of early stage of osteonecrosis of the femoral head. At present, ABR has proved to have good biocompatibility and bone conductivity in both animal experiments and clinical trials [10–13]. Due to the advantage of the angioconductive properties and their porosity for blood flow [10, 14], ABR is considered as a satisfactory artificial bone to fill the bone tunnel [15, 16]. However, ABR takes 4–8 weeks to complete vascularization and participate in new bone formation and metabolism [15]. During this time, the femoral head may continue to undergo necrosis due to the lack of blood flow and nutrients. In contrast, BBC has stem cell activity and can work rapidly after implantation to promote cell proliferation in the necrotic area of the femoral head. Therefore, we hypothesize that combining ABR and BBC is potentially beneficial to improve the success rate of hip preservation surgery. The objective of the study was to determine whether BBC and ABR grafting with ACD could improve functional outcomes and reduce the necessity of THA for patients with early-stage ANFH.

## Methods

### Study design

The study design was a prospective, randomized, comparative clinical trial. The study design was strictly performed in accordance with the ethical principles described in the Declaration of Helsinki 2013 Revision, and the design was approved by the Human Ethics Committee of Guangdong Provincial People’ s Hospital. Written informed consent was provided by the patients prior to their inclusion in the study. The experimental protocol was submitted to Chictr.org.cn, and the protocol number is ChiCTR2000039595.

According to the results of Sen et al. [17], a sample size of 22 hips per group is considered sufficient with a one-sided alpha level of 0.05, 80% power. Taking into account a lost to follow-up rate of about 10%, we planned to enroll a minimum size of 24 hips in each group.

### Patients

Patients who were eligible to participate in this study were recruited from the Center of Orthopedics Surgery from May 2015 to May 2020 by a designated surgeon. We confirmed the diagnosis of ANFH by examining the patient medical history, physical examination, and radiological tests [2].

The inclusion criteria were (1) patient age of 18 to 60 years old and (2) clear ANFH diagnosis (either unilateral or bilateral). The exclusion criteria were (1) < 18 or > 60 years old; (2) vascular disorders affecting lower limb function; (3) advanced ANFH with secondary arthritic bone changes and acetabular rim changes; (4) previous history of lower limb fractures, bone tumors, or other lesions; (5) inflammatory arthritis; (6) congenital deformity or insufficiency of lower limb; (7) infection in the surgical site; (8) lower limb surgery in the past 3 months; and (9) unwilling to undergo core decompression.

### Randomization

A statistician prepared a concealed, computer-generated, 1:1 randomization list. Randomization was performed by trained staff members using a parity distribution of the random numbers. The hips were randomly allocated to group A (received ACD with BBC and ABR grafting) and group B (received ACD with β-TCP granules and ABR grafting). Patients included in the study were assigned a sequential study number. A random allocation sequence was concealed by a staff member in consecutively numbered, opaque, sealed envelopes, and the staff member was not involved in the trial. Before surgery, an envelope containing the surgical plan for each hip was opened by a surgical assistant. The surgical assistant was not involved in the further follow-up of the patients.

### Surgical procedure

All surgical procedures were performed under either general or combined spinal anesthesia, and patients were in supine position on the traction table. Approximately, 30 to 50 ml of bone marrow was aspirated from the anterior superior iliac spine on one side of the patients using a bone marrow aspiration needle (Fig. 1a). The bone marrow was collected in the heparinized tubes and immediately centrifuged at 1500 rpm for 10 min (Eppendorf, AG 22331, Hamburg, Germany). After centrifugation, the bone marrow was divided into three layers (Fig. 1b). We collected 3 ml from the middle of the tube containing the enriched bone marrow cells with a 5-mL syringe [18]. Then, the subcutaneous tissue and periosteum were freed through a 2-cm longitudinal skin incision at the anterior superior iliac spine. A bone block with a volume of 2.0 × 2.0 × 0.5 cm medial to the ilium was removed and mechanically disaggregated into smaller pieces. The crushed bones were mixed with the bone marrow concentrate (Fig. 1c).

**Fig. 1:** **a** Bone marrow aspiration. **b** Bone marrow after centrifugation. **c** Mixture of crushed bones and BBC

For advanced core decompression, a 3-mm Kirschner wire was drilled by electric drill 2 cm below the greater trochanter, and the tip of Kirschner wire was placed in the necrotic area within the femoral head using C-arm fluoroscopy (Fig. 2a). With the K-wire as the center, the cannulated drill was used to drill a 12-mm bone channel over the Kirschner wire to release pressure in the femoral head (Fig. 2b). The blades at the tip of the bone reamer (Chinese Patent ZL 2009 1 0197369.5) can be expanded by turning the blade control knob at the end of the handle. After adjusting to the appropriate size, the blades can be rotated by turning the handle and the necrotic area removed by gradually increasing size of the blade (Fig. 2c).

**Fig. 2:** **a** Insertion of Kirschner wire. **b** Core decompression. **c** Necrosis removal. **d** Autologous bone and BBC grafting. **e** Insertion of the ABR

Finally, the necrotic area and the bone channel were backfilled. In group A, the mixture of autologous bone and BBC was introduced through the bone channel into the necrotic area of the femoral head and was tamped by a pestle (Fig. 2d). Then, the angioconductive bioceramic rod (ABR) was used to backfill the bone channel (Fig. 2e). In group B, the β-TCP granules (Fig. 3a) and ABR (Fig. 3b) were grafted and impacted successively. The entire process was conducted with sterile technique, and patients were allowed partial weight bearing with crutches for 3 months post-surgery.

**Fig. 3:** **a** β-TCP granules. **b** Angioconductive bioceramic rod (ABR)

### Outcome assessment

Preoperatively, the baseline information, including age, sex, weight, etiology, preoperative Ficat stage of ANFH, and Harris Hip Scores, was collected blindly. The Ficat stage of ANFH was determined according to the X-ray radiography of the hip. All participants received follow-up postoperatively. Harris Hip Scores (HHS) were used as the primary outcome of the study, and the rate of clinical failures of the operated hips at the last follow-up was used as the secondary outcome. In addition, pain and function scores were supplied by the pain and function components of HHS. Clinical failure was defined as the subsequent need to perform THA on patients.

### Statistical analysis

Data were analyzed using Statistical Package for Social Sciences (version 23.0; SPSS, Chicago, IL). The significance level was set at *P* value less than 0.05. Independent sample t test was used for the comparison of the means between the two groups. Categorical variables were compared by the Pearson chi-square test or Fisher exact test. All quantitative variables were depicted as mean and standard deviation. Survival was assessed using the Kaplan-Meier test and compared using a log-rank test.

## Results

### Baseline demographic characteristics

In all, 80 patients (100 hips) were initially recruited for this study. Among these, 36 patients (43 hips) were excluded and 44 patients (57 hips) met the study criteria and were enrolled. The selected candidates were randomly allocated into group A (received ACD with BBC and ABR grafting) and group B (received ACD with β-TCP granules and ABR grafting). During the 5-year follow-up period, 4 patients (6 hips) were lost (lost contact with patients), including 1 patient (2 hips) in group A and 3 patients (5 hips) in group B. In total, 40 patients (51 hips) were ultimately included for analysis (Fig. 4). The mean age was 37.70 ± 10.74 years (range 18 to 56 years) with no statistically significant difference between the two groups (*P* = 0.25) (Table 1). The baseline demographic characteristics of the current study subjects were homogeneous, and the mean follow-up time was 2 years.

**Fig. 4:** Flowchart of the study

**Table 1:** Baseline characteristics of the patients

Variable	Group A (*N* = 17)	Group B (*N* = 23)	*P* value
Number of hips	22	29	
Age, years	35.4 ± 11.1	39.4 ± 10.4	0.252
Sex			0.605
Male	12 (70.6%)	19 (82.6%)	
Female	5 (29.4%)	4 (17.4%)	
Weight (kg)	65.6 ± 14.7	65.3 ± 7.7	0.949
Hip involved unilateral	12 (70.6%)	17 (73.9%)	1.000
Hip involved bilateral	5 (29.4%)	6 (26.1%)	
Etiology			0.080
Steroid	8 (36.4%)	3 (10.3%)	
Alcohol	5 (22.7%)	9 (31.1%)	
Idiopathic	9 (40.9%)	17 (58.6%)	
Ficat stage			0.114
Stage I	1 (4.5%)	1 (3.4%)	
Stage II	19 (86.4%)	20 (69.0%)	
Stage III	2 (9.1%)	6 (20.7%)	
Stage IV	0 (0)	2 (6.9%)	
Pain scores	17.7 ± 4.3	17.6 ± 5.1	0.917
Function scores	49.5 ± 7.8	50.9 ± 9.0	0.550
Harris Hip Scores	67.2 ± 9.2	68.5 ± 13.1	0.678

Group A, bone marrow buffy coat graft group; group B, control group

### Functional outcomes

Preoperative pain scores, function scores, and HHS of the patients in both groups were not statically distinguishable. The mean postoperative pain scores were 31.8 ± 10.5 in group A and 26.9 ± 12.0 in group B at final follow-up (*P* = 0.133). The mean postoperative function scores were 52.3 ± 6.5 and 45.9 ± 13.9 in groups A and B, respectively, and this difference was statistically significant (*P* = 0.032). The mean postoperative Harris Hip Scores were 84.1 ± 14.2 and 72.8 ± 24.1 in groups A and B, respectively, at final follow-up with a statistically significant difference in the scores (*P* = 0.041) (Table 2). Fourteen (72.7%) hips in group A had a good to excellent outcome compared with thirteen (44.9%) hips in group B, as rated by the HHS (Table 2) (Fig. 5).

**Table 2:** Pain-related outcomes and functional outcomes after surgery

Variable	Group A (*N* = 17)	Group B (*N* = 23)	*P* value
Pain scores	31.8 ± 10.5	26.9 ± 12.0	0.133
Function scores	52.3 ± 6.5	45.9 ± 13.9	0.032*
Harris Hip Scores	84.1 ± 14.2	72.8 ± 24.1	0.041*
Overall evaluation			0.052
Excellent	10 (45.4%)	9 (31.1%)	
Good	6 (27.3%)	4 (13.8%)	
Medium	6 (27.3%)	11 (37.9%)	
Poor	0 (0)	5 (17.2%)	

Group A, bone marrow buffy coat graft group; group B, control group. Segments with significant statistical differences (*P < 0.05) between the groups were marked with an asterisk

**Fig. 5:** A 20-year-old female who was in group A receiving ACD, BBC, and ABR grafting with Ficat stage II osteonecrosis of the right hip (preoperative HHS 80.00; postoperative HHS 100.00). **a** Preoperative radiography. **b** Postoperative radiography. **c**–**f** One, 3, 6, and 12 months postoperative radiography

### Survivorship during follow-up

At the final follow-up, 1 patient (1 hip) in group A underwent THA after 15 months, while 3 patients (5 hips) in group B underwent THA after 6, 6, 9, 10, and 10 months (Table 3) (Figs. 6 and 7). The clinical failure rate was 4.5% (1/22) and 17.2% (5/29) in groups A and B, respectively, with a continuous correction chi-square test *P* value of 0.340 (Table 3). Kaplan-Meier analysis did not show obvious statistical differences in survival (*P* = 0.203) but suggested a trend that survivorship of the femoral head in group A is higher than that in group B (Fig. 8). Using Spearman’s rank correlation, there were correlations between the postoperative HHS and the conversion to hip arthroplasty.

**Table 3:** Number of patients receiving THA during the follow-up

Group	Group A (*N* = 17)		Group B (*N* = 23)		*P* value
Outcome	Hip preserved	THA	Hip preserved	THA	
Number of patients	16 (94.1%)	1 (5.9%)	20 (87.0%)	3 (13.0%)	0.624
Number of hips	21 (95.4%)	1 (4.5%)	24 (82.8%)	5 (17.2%)	0.340

Group A, bone marrow buffy coat graft group; group B, control group

**Fig. 6:** A failure case: a 49-year-old male who was in group B receiving ACD, β-TCP granules, and ABR grafting in the left hip. He had to perform THA 27 months later because of the failure of hip-preserving surgery. **a** Preoperative X-rays. **b** One month postoperative X-rays. **c** Twenty-seven months postoperative X-rays. **d**, **e** Computed tomography (CT) before THA. **f** Three-dimensional reconstruction based on CT before THA. **g**–**i** Magnetic resonance imaging (MRI) before THA

**Fig. 7:** Femoral head sample was collected for pathology examination and later analyses from the same patient in Fig. 6. **a** Gross morphology of the necrotic femoral head. **b** Tissue sections were imaged at × 10 magnification

**Fig. 8:** Kaplan-Meier survival curve showing the femoral head survival based on the different therapy

## Discussion

Based on the results of this prospective, randomized, and comparative study, the patient’s condition improved and symptoms were relieved in both groups after hip-preserving surgery and no patients experienced complications or adverse effects. In addition, patients in group A had higher postoperative function score (*P* = 0.032) and postoperative Harris Hip Scores (HHS) (*P* = 0.041) than patients enrolled in group B. The Kaplan-Meier survival analysis suggests that survival of the femoral head in group A is higher than that in group B.

The mean age of both A and B groups (35.4 vs. 39.4, respectively) in the present study was relatively young. However, most of the studies concerned with mid- to long-term prognosis of femoral head necrosis enroll patients with a similar mean age (24.7–42.0) [1], and the peak age incidence of femoral head necrosis is between 30 and 50 years. Thus, we propose that our study is representative. The relatively young age of the participants in our study is a potential explanation of the lower rate of hip arthroplasty, but this failed to reach a statistically significant difference. Moreover, we suggest that the relatively short follow-up time (mean follow-up time of 2 years) may influence these findings as it often requires 5–10 years for patients with femoral head necrosis to progress to end-stage hip disease [19].

CD is a common modality used in the treatment of early ANFH, but traditional CD has some limitations such as inadequate removal of the necrotic area. The clinical failure rates of CD have been reported to be between 20 and 70% [18]. Recently, advanced core decompression (ACD) has become more reliable and more common for the treatment for early stages of ANFH [20]. The difference between ACD and CD includes application of the expandable reamer which can expand the region of necrosis of the femoral head precisely and thoroughly. Lin et al. [21] reported that the single-blade expandable reamer has many strengths, and this technique is an effective hip-preserving surgery for early ANFH. In addition, another study showed that the first follow-up results of ACD are encouraging for early ANFH, especially the high stability of the femoral neck after ACD which allows quick rehabilitation [22]. In the present study, we used the bone reamer to remove the necrotic tissue, and bone grafts, through the ACD bone channel, to the necrotic area were used to enhance mechanical support and prevent collapse in the subchondral bone. Although the current form of ACD seems not meaningful in patients with a progressed lesions [22], we consider it technically easier to perform than a bone graft and has no additional risk.

MSCs are multipotent active cells with the capacity to differentiate into osteoblasts, most notably, the bone marrow-derived MSCs (BM-MSCs) with the superiority of bone and cartilage repair. Given this, MSCs are a promising and reliable approach for early ANFH. There are a large number of cytokines released by the BM-MSCs to promote angiogenesis, chondrogenesis, and osteogenesis, including vascular endothelial growth factor (VEGF), transforming growth factor-beta (TGF-β), and bone morphogenetic protein-2 (BMP2) [23–25]. Osteoprogenitor and vascular endothelial progenitor cells were filled into the necrotic area of the femoral head by providing BM-MSCs through the ACD bone channel to promote repair and regenerate bone tissue [26]. BBC or PRP for early-stage ANFH therapy has been confirmed as an effective strategy according to some studies [9, 18, 27–29]. In this study, patients receiving ACD, BBC, and ABR had a better primary outcome than the control group, but the overall difference was not statistically significant. The most likely reason for this outcome was that the follow-up duration was insufficient.

BBC was used as sources for the BM-MSCs because it was technically easy to obtain by centrifugation in an aseptic environment without ex vivo culture. Our previous studies had revealed that patients have greater benefit from BBC without large cost and additional risks [9, 18]. None of the patients who were implanted with BBC reported complications or adverse effects. BBC is rich in endothelial progenitors and hemangioblasts which promote angiogenesis in the necrotic area to facilitate revascularization. BBC also can improve the short-term functional outcomes, which is consistent with the results from a recent meta-analysis and systemic review of the data [6, 30, 31]. Therefore, due to the advantage of stem cell activity and easy accessibility, BBC is considered beneficial when combined with ACD to treat the ANFH.

This study has some limitations. First, it was a single-center study with a short period of study. Second, there were limited numbers of patients included in the final analysis, and this could affect the results. Third, blinding was not used because we considered it unethical to expose participants in the control group to the risks associated with incision in the anterior superior iliac spine. Fourth, the follow-up time was short (mean follow-up time = 2 years), and we plan to continue mid-term and long-term follow-up on patients in both study groups.

## Conclusion

Short-term follow-up results showed that the autologous bone marrow buffy coat and angioconductive bioceramic rod grafting with advanced core decompression is effective in the treatment of early ANFH. Data gathered also suggested a trend that the survivorship of the femoral head is higher for the patients receiving BBC and ABR with ACD.

## Data Availability

The data and materials used and/or analyzed during the current study are not publicly available but available from the corresponding authors on reasonable request.

## Abbreviations

ANFH: Avascular femoral necrosis of femoral head
ABR: Angioconductive bioceramic rod
BBC: Bone marrow buffy coat
ACD: Advanced core decompression
β-TCP: β-Tricalcium phosphate
CD: Core decompression
MSC: Mesenchymal stem cell
THA: Total hip arthroplasty
